The article "Efficacy of pentoxifylline treatment for neonatal sepsis: a meta-analysis of randomized controlled studies" was retracted in 2021. Reasons: plagiarism; overlap with other authors' work.

# Efficacy of pentoxifylline treatment for neonatal sepsis: a meta-analysis of randomized controlled studies

**DOI:** 10.1186/s13052-019-0697-8

**Published:** 2019-08-22

**Authors:** Jun Tian, Peifang Shen, Kaiyu Pan, Qiong Zhou

**Affiliations:** 1 Department of pediatrics, The First people’s Hospital of Xiaosha, Hangzhou, China; 2 Department of pediatrics, Children’s Hospital of Hangzhou, No 318 Chaowang Road, Hangzhou, 310005 Zhejiang Province People’s Republic of China

**Keywords:** Pentoxifylline, Neonatal sepsis, Mortality, Randomized controlled trials, Meta-analysis

## Abstract

**Introduction:**

Pentoxifylline may be an important approach to treat neonatal sepsis. However, its use has not been well established. We conduct a systematic review and meta-analysis to evaluate the efficacy of pentoxifylline treatment for neonatal sepsis.

**Methods:**

PubMed, Embase, and the Cochrane Central Register of Controlled Trials are searched. Randomized controlled trials (RCTs) assessing the influence of pentoxifylline treatment on neonatal sepsis are included. Two investigators independently have searched articles, extracted data, and assessed the quality of included studies. This meta-analysis is performed using the random-effect model.

**Results:**

Seven RCTs involving 439 patients are included in the meta-analysis. Compared with control intervention for neonatal sepsis, pentoxifylline treatment is associated with reduced hospital stay (Std. MD = -0.61; 95% CI = -0.93 to − 0.29; *P* = 0.0002) and metabolic acidosis (RR = 0.38; 95% CI = 0.22 to 0.66; *P* = 0.0006), but has no remarkable impact on mortality (RR = 0.59; 95% CI = 0.30 to 1.16; *P* = 0.13), serum TNF-α (Std. MD = -0.38; 95% CI = -1.29 to 0.52; *P* = 0.41), serum CRP (Std. MD = -0.25; 95% CI = -0.92 to 0.42; *P* = 0.47), plasma IL-6 (Std. MD = -0.13; 95% CI = -0.41 to 0.15; *P* = 0.37), disseminated intravascular coagulopathy (RR = 0.55; 95% CI = 0.25 to 1.21; *P* = 0.14), and oliguria/anuria (RR = 0.77; 95% CI = 0.28 to 2.16; *P* = 0.62). In addition, pentoxifylline treatment can significantly reduce mortality (RR = 0.50; 95% CI = 0.29 to 0.88; *P* = 0.02) after excluding the study conducted by Akdag during the sensivity analysis.

**Conclusions:**

Pentoxifylline treatment may be associated with reduced mortality and hospital stay in neonatal sepsis.

## Introduction

Neonatal sepsis is known as the most common cause of death in newborn infants, with the incidence of 6.5–38 among 1000 live births [1–3]. The combined rate of major morbidity and mortality of sepsis is up to 10–20% for all infants and 20–30% for very low birth weight infants [4–6]. Preterm infants with Gram-negative septic shock have the death rate of 65–85% despite of broad-spectrum antibiotics and intensive supporting care [7]. The morbidity and mortality may be caused by ineffective antibiotics to multidrug resistant bacteria or a weak host defense mechanisms in preterm infants [8–10].

The article "Efficacy of pentoxifylline treatment for neonatal sepsis: a meta-analysis of randomized controlled studies" was retracted in 2021. Reasons: plagiarism; overlap with other authors' work.

Adjuvant therapies may be increasingly important to increase the efficacy of antimicrobial agents and overcome excessive or uncontrolled inflammatory response in sepsis [11–13]. Redox-active agents (e.g. lactoferrin, zinc, selenium, ibuprofen, edaravone and pentoxifylline) have shown some efficacy to treat neonatal sepsis [14–17]. Pentoxifylline is a phosphodiesterase inhibitor among other actions, and can inhibit the production of tumor necrosis factor-alpha (TNF-α), preserve microvascular blood flow, prevent circulatory failure and intestinal vasoconstriction. It is reported to have beneficial effects on endothelial cell function and coagulation in sepsis, and the reduction of mortality from sepsis [18–20].

However, the use of pentoxifylline for neonatal sepsis has not been well established. Recently, several studies on the topic have been published, and the results have been conflicting [21–24]. Considering these inconsistent effects, we therefore conducted a systematic review and meta-analysis of RCTs to evaluate the efficacy of pentoxifylline treatment for neonatal sepsis.

## Materials and methods

Ethical approval and patient consent are not required since this is a systematic review and meta-analysis of previously published studies. The systematic review and meta-analysis are conducted and reported in adherence to PRISMA (Preferred Reporting Items for Systematic Reviews and Meta-Analyses) [25].

### Search strategy and study selection

Two investigators have independently searched the following databases (inception to June 2018): PubMed, Embase, and the Cochrane Register of Controlled Trials. The electronic search strategy is performed using with the following keywords: pentoxifylline, neonatal or infants or neonate, and sepsis. We also have checked the reference lists of the screened full-text studies to identify other potentially eligible trials.

The following inclusive selection criteria are applied: (i) population: neonatal sepsis; (ii) intervention: pentoxifylline treatment; (iii) comparison: matched placebo; and (iv) study design: RCT.

### Data extraction and outcome measures

We have used a piloted data-extraction sheet, which covers the following information: first author, number of patients, gestational age, male, birth weight, and detail methods in two groups. Data are extracted independently by two investigators, and discrepancies are resolved by consensus. We have contacted the corresponding author to obtain the data when necessary. No simplifications and assumptions are made.

The article "Efficacy of pentoxifylline treatment for neonatal sepsis: a meta-analysis of randomized controlled studies" was retracted in 2021. Reasons: plagiarism; overlap with other authors' work.

The primary outcome is mortality. Secondary outcomes include hospital stay, serum TNF-α, serum C-reactive protein (CRP), plasma interleukin (IL)-6, metabolic acidosis, disseminated intravascular coagulopathy, and oliguria/anuria.

### Quality assessment in individual studies

The Jadad Scale is used to evaluate the methodological quality of each RCT included in this meta-analysis [26]. This scale consists of three evaluation elements: randomization (0–2 points), blinding (0–2 points), dropouts and withdrawals (0–1 points). One point would be allocated to each element if they have been mentioned in article, and another one point would be given if the methods of randomization and/or blinding had been appropriately described. If the methods of randomization and/or blinding were inappropriate, or dropouts and withdrawals had not been recorded, then one point was deducted. The score of Jadad Scale varies from 0 to 5 points. An article with Jadad score ≤ 2 is considered to be of low quality. If the Jadad score ≥ 3, the study is thought to be of high quality [27].

## Statistical analysis

We have estimated standard mean differences (Std. MDs) with 95% confidence intervals (CIs) for continuous outcomes (hospital stay, serum TNF-α, serum CRP, and plasma IL-6), and risk ratios (RRs) with 95% CIs for dichotomous outcomes (mortality, metabolic acidosis, disseminated intravascular coagulopathy, and oliguria/anuria). A random-effects model is used regardless of heterogeneity. Heterogeneity is reported using the I^2^ statistic, and I^2^ > 50% indicates significant heterogeneity [28]. Whenever significant heterogeneity is present, we search for potential sources of heterogeneity. Sensitivity analysis is performed to detect the influence of a single study on the overall estimate via omitting one study in turn when necessary. Owing to the limited number (< 10) of included studies, publication bias is not assessed. Results are considered as statistically significant for *P* < 0.05. All statistical analyses are performed using Review Manager Version 5.3 (The Cochrane Collaboration, Software Update, Oxford, UK).

## Results

### Literature search, study characteristics and quality assessment

A detailed flowchart of the search and selection results is shown in Fig. 1. 719 potentially relevant articles are identified initially. Finally, seven RCTs that meet our inclusion criteria are included in the meta-analysis [20–24, 29, 30].

**Fig. 1:** Flow diagram of study searching and selection process

The main characteristics of the seven included RCTs are presented in Table 1. The seven studies are published between 1996 and 2015, and sample sizes range from 20 to 120 with a total of 439. Pentoxifylline is administered by 5–6 mg/kg/h intravenously for 4-6 h daily, and the duration time ranges from 3 days to 6 days.

The article "Efficacy of pentoxifylline treatment for neonatal sepsis: a meta-analysis of randomized controlled studies" was retracted in 2021. Reasons: plagiarism; overlap with other authors' work.

**Table 1:** Characteristics of included studies

NO.	Author	Pentoxifylline group					Control group					Jada scores
		Number	Gestational age (weeks)	Male (n)	Birth weight (g)	Methods	Number	Gestational age (weeks)	Male (*n*)	Birth weight (g)	Methods	
1	Shabaan 2015 [21]	60	30.2 ± 2.5	34	1404 ± 417	intravenous pentoxifylline 5 mg/kg/hr. for 6 h on 6 successive days	60	30.1 ± 2.2	44	1370 ± 471	matched placebo	5
2	Akdag 2014 [22]	51	31 (24–42)	29	1490 (620–4580)	pentoxifylline 6 mg/kg/h intravenously, over 4 h, daily for three consecutive days	51	31 (25–40)	33	1410 (620–4300)	matched placebo	4
3	Adel 2010 [23]	17	35.94 ± 4.04	9	2470 ± 890	pentoxifylline 5 mg/kg/h for 6 h, for 6 successive days	20	36.05 ± 3.2	11	2210 ± 590	matched placebo	4
4	Ali 2006 [24]	25	32–37	–	950–2580	pentoxifylline 5 mg/kg/h for 6 h, for 3 successive days	25	32–37	–	1000–2650	matched placebo	3
5	Selim 2004 [29]	13	37.62 ± 2.43	–	2509 ± 549	initiately 0.5 h before beginning antibiotic therapy and given in a dose of 0.5 mg/kg/h by continuous infusion for 24 h	7	38 ± 2.08	–	2822 ± 637	matched placebo	
6	Lauterbach 1999 [30]	40	31.6 ± 2.9	23	1690.2 ± 396.5	pentoxifylline 5 mg/kg/h for 6 h, for 6 successive days	38	32.8 ± 3.01	20	1749.8 ± 475.6	matched placebo	
7	Lauterbach 1996 [20]	16	31.54 ± 31	–	1752.09 ± 483.4	pentoxifylline 5 mg/kg/h for 6 h, for 3 successive days	16	32.35 ± 33	–	1861.29 ± 511.7	matched placebo	

Among the seven RCTs, six studies have reported mortality [20–24, 30], two studies have reported hospital stay [21, 23], three studies have reported serum TNF-α and serum CRP [21, 22, 29], three studies have reported plasma IL-6 [22, 29, 30], two studies have reported metabolic acidosis [21, 30], four studies have reported disseminated intravascular coagulopathy [21–23, 30], and four studies have reported oliguria/anuria [21–23, 30]. Jadad scores of the seven included studies vary from 3 to 5, and all seven studies are considered to be high-quality ones according to quality assessment.

### Primary outcome: mortality

This outcome data is analyzed with the random-effects model, and the pooled estimate of the six included RCTs suggested that compared to control group for neonatal sepsis, pentoxifylline treatment has no significant influence on mortality (RR = 0.59; 95% CI = 0.30 to 1.16; *P* = 0.13), with low heterogeneity among the studies (I^2^ = 30%, heterogeneity *P* = 0.21, Fig. 2).

**Fig. 2:** Forest plot for the meta-analysis of mortality

The article "Efficacy of pentoxifylline treatment for neonatal sepsis: a meta-analysis of randomized controlled studies" was retracted in 2021. Reasons: plagiarism; overlap with other authors' work.

### Sensitivity analysis

Low heterogeneity is observed among the included studies for the primary outcome. As shown in Fig. 2, the study conducted by Akdag shows the results that are almost out of range of the others and probably contribute to the heterogeneity [22]. After excluding this study, the results suggests that pentoxifylline treatment can significantly reduce mortality (RR = 0.50; 95% CI = 0.29 to 0.88; *P* = 0.02), and there is no heterogeneity among the remaining RCTs (I^2^ = 0%, heterogeneity *P* = 0.44).

### Secondary outcomes

Compared to control group for neonatal sepsis, pentoxifylline treatment is associated with remarkably decreased hospital stay (Std. MD = -0.61; 95% CI = -0.93 to − 0.29; *P* = 0.0002; Fig. 3), but shows no significant impact on serum TNF-α (Std. MD = -0.38; 95% CI = -1.29 to 0.52; *P* = 0.41; Fig. 4), serum CRP (Std. MD = -0.25; 95% CI = -0.92 to 0.42; *P* = 0.47; Fig. 5), plasma IL-6 (Std. MD = -0.13; 95% CI = -0.41 to 0.15; *P* = 0.37; Fig. 6). In addition, metabolic acidosis in pentoxifylline group is lower than that in control group (RR = 0.38; 95% CI = 0.22 to 0.66; *P* = 0.0006; Fig. 7). There is no significant difference of disseminated intravascular coagulopathy (RR = 0.55; 95% CI = 0.25 to 1.21; *P* = 0.14; Fig. 8), and oliguria/anuria (RR = 0.77; 95% CI = 0.28 to 2.16; *P* = 0.62; Fig. 9) between two groups.

**Fig. 3:** Forest plot for the meta-analysis of hospital stay (days)

**Fig. 4:** Forest plot for the meta-analysis of serum TNF-α

**Fig. 5:** Forest plot for the meta-analysis of serum CRP

**Fig. 6:** Forest plot for the meta-analysis of plasma IL-6

**Fig. 7:** Forest plot for the meta-analysis of metabolic acidosis

**Fig. 8:** Forest plot for the meta-analysis of disseminated intravascular coagulopathy

**Fig. 9:** Forest plot for the meta-analysis of oliguria/anuria

## Discussion

Strong and expensive antimicrobials agents have been extensively developed, but the mortality and morbidity of infants with sepsis are still high [21, 31, 32]. Adjuvant therapies using pentoxifylline have gained the great interest in clinical work [14]. Pentoxifylline is a nonsteroidal immunomodulating agent with unique hemorrheologic effects, and has been used in kinds of infectious, vascular and inflammatory diseases in children because of its potent anti-inflammatory properties through downregulation of proinflammatory cytokines and blood viscosity, and the increase in microcirculation and tissue perfusion [22, 29]. The current evidence is weakened, the routine use of pentoxifylline in neonatal sepsis has not been recommended.

One RCT has report that pentoxifylline has no influence on mortality in preterm infants with suspected or confirmed sepsis [21]. In contrast, significant reduction of mortality is observed in infants receiving pentoxifylline in other studies [24, 30]. One recent Cochrane review includes six small RCTs and quasi-RCTs, and reveals a significant reduction in all-cause mortality during hospital stay in neonates with sepsis after the use of pentoxifylline as an adjunct to antibiotics [33]. Our meta-analysis has included seven RCTs involving 439 neonates, and the results demonstrate that pentoxifylline has no substantial impact on mortality for neonatal sepsis, but is associated with significantly reduced hospital stay.

The article "Efficacy of pentoxifylline treatment for neonatal sepsis: a meta-analysis of randomized controlled studies" was retracted in 2021. Reasons: plagiarism; overlap with other authors' work.

TNF-α, IL-1 and IL-6 concentrations can be elevated in preterm infants with sepsis, and their high concentrations of those cytokines are associated with high mortality [34]. TNF-α, CRP and IL-6 do not differ between pentoxifylline group and control group based on the results of our meta-analysis. In addition, pentoxifylline treatment is associated with significantly reduced metabolic acidosis, but with no impact on disseminated intravascular coagulopathy and oliguria/anuria. Regarding the sensitivity analysis, significant reduction of mortality is found in pentoxifylline group compared to that in control group after excluding the study conducted by Akdag [22] (RR = 0.50; 95% CI = 0.29 to 0.88; *P* = 0.02), and there is no heterogeneity among the remaining RCTs. That study reports 24 mg/kg pentoxifylline daily, and other included RCTs report 30 mg/kg pentoxifylline daily. This heterogeneity may be attributed to the different doses of pentoxifylline use daily. In addition, the differences of mortality is reported to be possibly caused by different study populations related to the causative organisms of neonatal sepsis, but a subgroup analysis of pentoxifylline effect on infants’ mortality and short-term morbidity shows no significant difference in Gram-negative and Gram-positive sepsis groups [22].

This meta-analysis has several potential limitations that should be taken into account. First, our analysis is based on only seven RCTs, and five of them have a small sample size (*n* < 100). Overestimation of the treatment effect is more likely in smaller trials compared with larger samples. Next, the heterogeneity of mortality in this meta-analysis is possibly caused by different doses and methods of pentoxifylline treatment. Finally, some unpublished and missing data may lead bias to the pooled effect.

## Conclusion

Pentoxifylline treatment may provide some benefits to neonates with sepsis.

## Data Availability

Not applicable.

## Abbreviations

RCT: Randomized controlled trial
Std. MD: Standard Mean difference
RRs: risk ratios
CRP: C-reactive protein
